# TRIM65 Promotes Malignant Cell Behaviors in Triple-Negative Breast Cancer by Impairing the Stability of LATS1 Protein

**DOI:** 10.1155/2022/4374978

**Published:** 2022-08-17

**Authors:** Yongbin Lu, Yi Xiao, Jingru Yang, Hongxin Su, Xiaobin Zhang, Fei Su, Baohong Tian, Da Zhao, Xiaoling Ling, Tao Zhang

**Affiliations:** ^1^Department of Oncology, The First Hospital of Lanzhou University, Lanzhou, China; ^2^College of Earth and Environmental Sciences, Lanzhou University, Lanzhou, China; ^3^Scientific Development and Planning Department, The First Hospital of Lanzhou University, Lanzhou, China; ^4^Breast surgery, The First Hospital of Lanzhou University, Lanzhou, China; ^5^Department of Radiotherapy, The First Hospital of Lanzhou University, Lanzhou, China

## Abstract

TNBC is a malignant tumor that easily relapses and metastasizes, with a poor prognosis in women. Ubiquitination plays a key role in promoting the tumor process. In various tumors, TRIM65 can affect malignant biological tumor behavior by ubiquitination of related proteins. We aimed to investigate TRIM65 expression in TNBC and whether it promotes malignant biological behavior in TNBC cells using Cell Counting Kit-8, colony formation, and transwell assays. Mechanically, we confirmed that TRIM65 promoted TNBC invasion and metastasis by ubiquitination of LATS1 protein through Co-IP, CHX, and endogenous ubiquitination experiments. The expression of TRIM65 was abnormally high and accelerated the proliferation, invasion, and migration of MDA-MB-231 and MDA-MB-453 cells. *In vivo* animal experiments also revealed that TRIM65 accelerated TNBC cell proliferation. Mechanistically, TRIM65 degraded LATS1 protein expression through ubiquitination in the Co-IP, CHX, and endogenous ubiquitination experiments. Rescue assays confirmed that TRIM65 degraded LATS1 protein expression, accelerating the proliferation, invasion, and migration ability of TNBC cells. Our results show that TRIM65 is upregulated in TNBC, and TRIM65 degrades LATS1 protein expression through ubiquitination and promotes malignant biological behavior in TNBC cells. TRIM65 may play an important role as a new oncogene in TNBC.

## 1. Introduction

Breast cancer is one of the most critical health threats faced by women, and its incidence and prevalence increase daily [1]. In terms of the expression of biomarkers such as estrogen receptor, progesterone receptor, and human epidermal growth factor receptor 2 (HER2), breast cancer can be divided into the luminal A, luminal B, HER-2 overexpression, and triple-negative breast cancer (TNBC) types [2]. TNBC accounts for about 15%–20% of breast cancer cases and is prone to recurrence and metastasis, with a median overall survival rate of approximately 13 months [2]. Lifestyle and environmental factors have important impacts on TNBC progression, and the development of molecular events such as abnormal expression of cell oncogenes, enhanced invasion and migration ability, and blocked apoptosis have also promoted the occurrence and development of TNBC [3–5]. Although surgery, radiotherapy and chemotherapy, endocrine therapy, and other methods have improved the treatment effect and survival time for patients with TNBC, these patients are prone to relapse and metastasis, and the prognosis is poor [6, 7]. Therefore, there is an urgent need for researchers to identify effective therapeutic targets and carry out molecular targeted therapies for TNBC.

One known mechanism of TNBC includes an ubiquitination process, which usually requires the E1 ubiquitin-activating enzyme, E2 ubiquitin-conjugating enzyme, and E3 ubiquitin ligase. E3 ubiquitin ligase binds ubiquitin to protein substrates and plays a special role in the regulation of ubiquitin [8]. Tripartite motif containing 65 (TRIM65) belongs to the triple motif protein family [9], which is mainly composed of a RING finger domain, one or two B-box domains, a helix-helix domain, and a highly diverse C-terminal domain. RING is a cysteine-rich zinc binding domain with E3 ubiquitin ligase activity [9]. TRIM65 was originally found to be a genetic polymorphism associated with white matter lesions [10], and subsequent research found that TRIM65 was abnormally highly expressed in many types of cancer, including lung [11], liver [12], bladder [13], and glioma [14]. However, there are no reports on the differential expression of TRIM65 in breast cancer. As an E3 ubiquitin ligase, TRIM65 is involved in ubiquitination in a large number of cancers. Yang et al. have previously found that TRIM65 accelerates the proliferation and metastasis of liver cancer cells by ubiquitinating Axin1 and activating *β*-catenin signaling [12]. Similarly, Hu et al. showed that TRIM65 overexpression plays a carcinogenic role in the pathogenesis of glioma through ANX2 ubiquitination and may be used as a new therapeutic target for glioma [14]. TRIM65 has also been shown to promote colorectal cancer metastasis through targeted ubiquitination and degradation of ARHGAP35 protein [15] and activates ERK1/2/C-myc signaling by targeting ubiquitination to degrade DUSP6 protein, thereby promoting the invasion of endometrial stromal cells [16]. Ubiquitination plays a vital role in promoting the development of breast cancer [17, 18]. In breast cancer specifically, Guo et al. found that TRIM31 promotes progression through ubiquitination and degradation of the K48 and K63 sites of p53 [19], and Zhang et al. showed that TRIM7 regulates the migration and invasion of osteosarcoma cells through ubiquitination of a breast cancer metastasis inhibitor [20].

To our knowledge, no association between TRIM65 and breast cancer or TNBC has been reported in any previous studies. We hypothesized that TRIM65 was abnormally high in TNBC and promotes the invasion and metastasis of TNBC cells *in vitro* and *in vivo* experiments. We aimed to identify the mechanism by which TRIM65 degrades large tumor suppressor kinase 1 (LATS1) protein expression and promotes the invasion and metastasis of TNBC cells through ubiquitination using coimmunoprecipitation (Co-IP), cycloheximide (CHX), and endogenous ubiquitination experiments. Compared with previous studies on TNBC, our study for the first time found high expression of TRIM65 in TNBC and with poor prognosis and proved for the first time that TRIM65 promotes TNBC through ubiquitin LATS1. This study is expected to find a new therapeutic target for TNBC patients and provide a new theoretical and experimental basis for clinical treatment. Considering that TRIM65 promotes LATS1 degradation, our next goal will be to further study whether TRIM65 degradation depends on its catalytic activity using truncation and mutation experiments and explore the influence of LATS1 binding and LATS1 degradation on the main downstream pathways.

## 2. Materials and Methods

### 2.1. Cell Culture

Human breast cancer cell lines which included BT-549, MDA-MB-231, MDA-MB-453, and MCF-10A were obtained from American Type Culture Collection (Manassas, VA, USA). All cells were maintained in the Roswell Park Memorial Institute 1640 medium (Gibo, Grand Island, NY, USA) or Dulbecco's modified Eagle's medium (Gibco, Grand Island, NY, USA) supplemented with 10% fetal bovine serum (10% v/v, Gibco, Grand Island, NY, USA) in a humidified atmosphere of 5% CO_2_ at 37°C according to the manufacturer's protocol. Cells were seeded onto 96-well plates at a density of 3–5 × 10^3^/well.

### 2.2. Lentivirus Infection

Short hairpin RNA (shRNA) against TRIM65 (sh-TRIM65) was based on the TRIM65 sequence listed in GenBank (NC_000017.11) and full-length sequence of LATS1 (NM_001270519.2). The psPAX2 and pMD2.G vector were obtained from Dianxi Bio Co., Ltd (Shanghai, China). An empty plasmid was used as the control (sh-NC). The cells (2 × 10^5^ cells/well) were seeded in a 24-well plate, cultured to 70% confluency, incubated with 2 *μ*g/*μ*L puromycin, and transfected with lentiviral vectors (1 × 10^5^ TU) for 48 h. We used the following shRNA sequences: NC, 5′-GCAAGCTGACCCTGAAGTT-3′; sh-TRIM65, 5′-GCTACAGGCCCTGGAAATA-3′; and sh-LATS1, 5′-GCAATCAGTTAACCGCAAA-3′. Efficiency was verified by quantitative real-time polymerase chain reaction (RT-qPCR) and Western blotting (WB).

### 2.3. Quantitative Real-Time Polymerase Chain Reaction

Total RNA was extracted from tissues or cells using TRIzol reagent (Life Technologies, Scotland, UK) according to the manufacturer's instructions. Reverse transcription was performed using Prime Script RT Master Mix (TaKaRa, Shiga, Japan). RT-qPCR was amplified using SYBR Select Master Mix (Applied Biosystems, Foster, CA, USA) and detected using the ABI 7500 sequencing system. GAPDH served as a loading control. The primer sequences are described as follows: TRIM65, forward, 5′-AAGCAGCCAGATCCAGAACTC-3′ adn reverse, 5′-ACAAACTGTGCTTGGGACCG-3′; GAPDH forward, 5′-AATGGGCAGCCGTTAGGAAA-3′ and reverse, 5′-GCGCCCAATACGACCAAATC-3′; and LATS1 forward, 5′-GATCCTCGACGAGAGCAGATG-3′ and reverse, 5′-CGTTGCTAGGGTGAGCTTGA-3′.

### 2.4. Western Blot

Total protein was prepared using the RIPA buffer (Invitrogen, Thermo Fisher Scientific, Waltham, MA, USA). The proteins were separated by 10% sodium dodecyl sulfate polyacrylamide gel electrophoresis and transferred to polyvinylidene fluoride membranes. Skimmed milk (5%) was blocked at room temperature for 1 h. Next, the membranes and primary antibodies were incubated overnight at 4°C. They were then incubated with secondary antibodies at room temperature for 1 h. Finally, the proteins were identified using enhanced chemiluminescence reagents (Thermo Fisher Scientific) using an enhanced chemiluminescence detection system. GAPDH served as a loading control for total proteins. The primary antibodies used were as follows: TRIM65 (ab165884, Abcam, Cambridge, MA, USA; 1 : 1000 dilution), LATS1 (ab70562, Abcam, Cambridge, MA, USA; 1 : 1000 dilution), LATS2 (ab110780, Abcam, Cambridge, MA, USA; 1 : 1000 dilution), GAPDH (ab181602, Abcam, Cambridge, MA, USA; 1 : 5000 dilution), and ubiquitin (ab7780, Abcam, Cambridge, MA, USA; 1 : 1000 dilution).

### 2.5. Cell Proliferation Analysis

Cells (5 × 10^3^/well) were seeded in 96-well plates. Ten microliters of Cell Counting Kit-8 (CCK-8) reagent (Dojindo Laboratories, Kumamoto, Japan) was added to evaluate cell proliferation every day in accordance with the manufacturer's instructions. The absorbance was measured at 450 nm using a spectrophotometer (Bio-Rad Laboratories, Hercules, CA, USA).

### 2.6. Liquid Chromatography with Tandem Mass Spectrometry Analysis

MDA-MB-231 after TRIM65 knockout was inoculated into a 10 cm petri dish, cultured for 24 h, washed by phosphate-buffered saline, and quenched by liquid nitrogen. Cells were collected with an extraction agent and washed by chloroform, and the supernatant was taken to a resting place. After sealing with a sealing membrane, the cells were stored in a refrigerator at at –80°C until analysis. The expression of other differentially expressed proteins was detected by liquid chromatography with tandem mass spectrometry (LC-MS/MS) (Agilent 6490, Agilent Technologies, Inc., Santa Clara, CA, USA) [21], and the top 10 differentially expressed proteins were selected for cluster analysis.

### 2.7. Coimmunoprecipitation

Cell lysates were prepared using lysis buffer (Pierce, Rockford, IL, USA). Lysates were centrifuged and cleared by incubation with protein A/G magnetic beads (Thermo Fisher Scientific) for 1-2 h at 4°C. The precleared supernatant was subjected to immunoprecipitation using the primary antibody LATS1 (ab70561, Abcam; 1 : 200) at 4°C overnight. The next day, the complexes were incubated with protein A/G magnetic beads for 1-2 h. Proteins were subsequently analyzed using WB [22].

### 2.8. *In Vitro* Ubiquitination Assay

MDA-MB-231 and MDA-MB-453 cells were treated with CHX (10 *μ*g/ml) after TRIM65 knockout. Cells were collected and treated for 0, 2, 4, and 6 h, and the protein expression of LATS1 cells was detected by WB. MDA-MB-231 and MDA-MB-453 cells were also treated with MG132 after TRIM65 knockout. After 24 hours, ubiquitinated proteins were captured by a nickel column, and the protein expressions of TRIM65 and LATS1 were detected by WB [23].

### 2.9. Cell Migration and Invasion Assays

Cells containing serum-free medium (3 × 10^4^/well) were added to the upper chamber of the transwell and stroma-coated (25 *μ*g, BD Biosciences) for invasion assay or Matrigel and inserted uncoated for migration assay. Subsequently, 600 *μ*L complete medium was added to the lower chamber of the transwell and incubated for 24 h. Finally, 4% paraformaldehyde was used for fixation, and 0.1% crystal violet was used for color rendering.

### 2.10. Immunohistochemistry (IHC)

The wax block specimens collected in advance were prepared into sections and added to xylene for dewaxing treatment. 1.5% H_2_O_2_ was added to the sections, and the samples were incubated with primary antibody at 4°C overnight (TRIM65, 1:250 and Ki67, 1:100). The next day, secondary antibody was added; DAB chromogenic reagent was added and counterstained with hematoxylin. The staining was observed under the microscope. The positive expression of TRIM65 is based on the appearance of brown-yellow particles in the cytoplasm, and those without coloration are negative. A semiquantitative scoring system was used to evaluate the staining effect. The TRIM65 dyeing intensity was scored as follows: 0 points (colorless), 1 point (weak dyeing, light yellow), 2 points (medium dyeing, brownish yellow), and 3 points (strong dyeing, brownish brown); the dyeing range was as follows: 0 points (≤20%), 1 point (21%–50%), 2 points (51%–80%), and 3 points (>80%). The product of the staining intensity score and the staining range score is the staining index. Staining index ≥ 2 is a positive expression, and <2 is a negative expression. Ki67 color index ≥ 10% is high expression, and <10% is low expression. All TNBC samples were obtained from the First Hospital of Lanzhou University. All experimental studies were approved by the ethics committee of the First Hospital of Lanzhou University (LDYYLL-2021-414).

### 2.11. Animal Models

Twelve immunodeficient female nude mice aged 4-5 weeks were purchased and randomly divided into two groups. All female nude mice were bred and tested according to the guidelines of the Animal Management Regulations of the First Hospital of Lanzhou University. We inoculated 10 × 10^7^ MDA-MB-231 and small interfering-TRIM65 MDA-MB-231 cells subcutaneously in nude mice of both groups; tumor length and width were measured periodically. After approximately 6 weeks, the nude mice were sacrificed. The tumor tissues were removed, weighed, measured, and stained with hematoxylin and eosin (H&E). Ki67 staining and cell proliferation were detected. The female nude mouse research protocol was authorized by the ethics committee of the First Hospital of Lanzhou University (LDYYLL-2021-414).

### 2.12. Statistical Analysis

Three replicates were performed for each experiment, and all data are reported as the mean ± standard error of the mean. All data were analyzed using a two-sided *t*-test. Related graphics were drawn using GraphPad Prism version 7.0. *p* < 0.05, *p* < 0.01, and *p* < 0.001 were considered statistically significant and are expressed as ^∗^, ^∗∗^, and ^∗∗∗^, respectively. *p* > 0.05 is expressed as n.s.

## 3. Results

### 3.1. TRIM65 Is Upregulated and Is an Independent Risk Factor for the Prognosis of TNBC

Based on our analysis of The Cancer Genome Atlas database, we found that TRIM65 was significantly upregulated in TNBC, and high expression of TRIM65 significantly reduced the overall survival risk of patients with TNBC (Figures 1(a) and 1(b)). Further univariate and multivariate analyses found that TRIM65 was an independent risk factor for the prognosis of TNBC; hazard ratios (95% confidence interval) were 1.95 (1.03–3.68) and 2.51 (1.20–5.25), respectively (Figures 1(c) and 1(d)).

Representative images and IHC analysis showed that TRIM65 was upregulated in patients with TNBC (Figures 2(a) and 2(b)). Compared with the adjacent tissues, TRIM65 was upregulated in TNBC tissues as demonstrated by WB analysis (Figure 2(c)). Furthermore, TRIM65 was upregulated in BT-549, MDA-MB-231, and MDA-MB-453 cells compared to MCF10A cells (Figure 2(d)).

### 3.2. TRIM65 Promotes Malignant Biological Behavior in TNBC Cells *In Vitro* and *In Vivo*

The efficiency of lentiviral constructs was calculated by RT-qPCR and WB analysis, and the results showed that TRIM65 mRNA and protein were significantly downregulated in the sh-TRIM65 group compared with the normal control (NC) group (Figures 3(a) and 3(b)). Subsequently, we performed cell phenotypic analysis. CCK-8 and colony-forming assays revealed that cell proliferation was suppressed in the sh-TRIM65 group compared with the NC group in MDA-MB-231 and MDA-MB-453 cells (Figures 3(c) and 3(d)). The transwell assay showed that cell invasion and migration were suppressed in the sh-TRIM65 group compared with the NC group in MDA-MB-231 and MDA-MB-453 cells (Figure 3(e)). The above results indicated that upregulated TRIM65 expression promotes malignant biological behavior in TNBC cells.

To further clarify the effect of TRIM65 on TNBC formation *in vivo*, we used a subcutaneous xenograft tumor model to study the effect of TRIM65 on TNBC (Figure 4(a)). We planted an equal number of cells in the NC and sh-TRIM65 groups under the skin of female immunodeficient mice. By examining the tumor size, growth curve, and tumor weight, we found that the volume and weight of TNBC tumors were significantly lower after 6 weeks in the sh-TRIM65 group than in the NC group. The results showed that knockdown of TRIM65 lowered tumor weight and volume in mice (Figures 4(b) and 4(d)). In the IHC analysis, the H&E stain and Ki67 of the sh-TRIM65 group were significantly higher than those of the NC group (Figures 4(e) and 4(f)). These results revealed that the upregulated expression of TRIM65 significantly promoted the tumorigenic ability of TNBC cells *in vivo*.

### 3.3. TRIM65 Accelerates Ubiquitin-Mediated LATS1 Protein Degradation

To explore the downstream-regulated target genes of TRIM65, the applicant conducted proteomics testing by LC-MS/MS after inhibiting the expression of TRIM65 in MDA-MB-231 cells and found that 43 proteins were downregulated and 74 were upregulated. The heat map shows the top 10 upregulated and downregulated proteins (Figure 5(a)). Subsequently, we analyzed the correlation between TRIM65 and LATS1 and LATS2 using the StarBase database and found that TRIM65 was correlated with LATS1 but not with LATS2, with correlation coefficients (*r*) of -0.215 and -0.069, respectively (Figure 5(b)). To understand whether TRIM65 regulates the expression of LATS1, we conducted further analyses through WB experiments. The results showed that the sh-TRIM65 group showed increased expression of LATS1 but not LATS2 in MDA-MB-231 and MDA-MB-453 cell lines (Figure 5(c)). These results proved that TRIM65 regulates the expression of LATS1.

To investigate whether TRIM65 regulates LATS1 at the transcriptional or posttranscriptional level, we performed RT-qPCR assays. The results showed no substantial changes in LATS1 transcript levels, while TRIM65 was silenced (Figure 6(a)). We then performed Co-IP assays on MDA-MB-231 and MDA-MB-453 cells. TRIM65 was found in complexes with antibodies against LATS1 in both cell lines (Figure 6(b)), which indicated an *in vivo* binding between LATS1 and TRIM65 in MDA-MB-231 and MDA-MB-453 cells. Next, we used the protein synthesis inhibitor CHX in subsequent experiments. WB was performed in the presence of CHX after 6 h, showing that the knockdown of TRIM65 inhibited LATS1 degradation in TNBC cells (half-life, ~4 h vs. >6 h, MDA-MB-231-NC and MDA-MB-231-sh-TRIM65 and <4 h vs. >4 h, MDA-MB-453-NC and MDA-MB-453-sh-TRIM65; Figure 6(c)). In addition, at 6 h, the sh-TRIM65 group retained more LATS1 protein expression. Endogenous LATS1 ubiquitination was reduced in MDA-MB-231/MDA-MB-453-sh-TRIM65 cells compared to the NC group, and protein expression of LATS1 was increased (Figure 6(d)). Collectively, TRIM65 augments ubiquitin-mediated degradation of the LATS1 proteins.

### 3.4. TRIM65 Promotes Malignant Biological Behavior by Degrading LATS1 Expression in TNBC Cells

Finally, in the NC group, the sh-TRIM65, sh-TRIM65, and sh-LATS1 cotransformation groups were constructed for rescue experiments in MDA-MB-231 and MDA-MB-453 cell lines. Compared with the NC group, CCK-8 and colony formation assays indicated that the cell proliferation ability of TNBC cells was decreased in the sh-TRIM65 and cotransfer groups. Compared with sh-TRIM65, the impaired proliferation ability of TNBC was partially recovered in the cotransfer group in MDA-MB-231 and MDA-MB-453 cells (Figures 7(a) and 7(b)). Compared with the NC group, the transwell assay indicated that the invasion and migration abilities of TNBC cells in the sh-TRIM65 and cotransfer groups were reduced. Compared with the sh-TRIM65 group, the invasion and migration ability of TNBC cells were improved, and the impaired invasion and migration abilities were partially recovered in the cotransfer group in MDA-MB-231 and MDA-MB-453 cells (Figure 7(c)). TRIM65 degrades the expression of LATS1 protein through ubiquitination, thereby promoting malignant biological behavior in TNBC cells (Figure 7(d)).

## 4. Discussion

Female breast cancer has surpassed lung cancer and ranks first among new tumors. Patients with breast cancer comprised 2.3 million new cases of cancer in 2020, accounting for approximately 11.7% of all tumors [1]. TNBC is the most aggressive type of breast cancer and is difficult to cure [24]. Hence, it is imperative to explore the molecular mechanism of TNBC and seek molecular targeted therapy for early TNBC.

TRIM65 belongs to the ubiquitin E3 ligase family and plays an important role in developmental disorders, viral infections, and cancer [11–14, 25]. Studies have shown that TRIM65 is a potential carcinogen in the pathogenesis of bladder cancer, and TRIM65 overexpression is an independent prognostic factor for bladder cancer [13]. TRIM65 acts as an oncogene in hepatocellular carcinoma, and its high expression promotes cancer cell proliferation and metastasis in liver cancer tissue [12]. Our results showed that TRIM65 was highly upregulated and was an independent prognostic factor in TNBC. After inhibiting the expression of TRIM65, the proliferation, invasion, and migration of TNBC cells were significantly inhibited in MDA-MB-231 and MDA-MB-453 cells. *In vivo* experiments showed that inhibiting the expression of TRIM65 can also inhibit the growth of tumor cells, which is consistent with the *in vitro* experiments.

Epigenetic modifications such as methylation, acetylation, and ubiquitination are important research fields, as they affect oncogene overexpression or tumor suppressor gene silencing, thereby stimulating tumorigenic pathways and influencing TNBC treatment [26, 27]. TRIM65 acts as an E3 ubiquitinated ligase as a targeted regulatory substrate in various tumors to promote tumorigenesis and development. TRIM65 accelerates colorectal cancer metastasis by targeted degradation of ARHGAP35 protein [15], promotes the invasion of endometrial stromal cells through DUSP6 ubiquitination, activates ERK1/2/C-myc signals [16], and promotes bladder cancer cells through ubiquitination and degradation of ANXA2 invasion [13].

To identify the protein that interacts with TRIM65, we used proteomic analysis to determine whether TRIM65 protein can interact with LATS1. When TRIM65 was knocked down, the protein expression of LATS1 was significantly upregulated. We found that TRIM65 expression was significantly negatively correlated with LATS1 (correlation coefficient *r* = −0.215). Furthermore, we knocked down TRIM65, and WB showed that the expression of LATS1 protein increased, although no effect was observed on LATS2. We then used the Co-IP method to detect whether TRIM65 specifically interacts with LATS1, and the results showed that TRIM65 binds to LATS1 protein. Through CHX experiments, we found that the downregulation of TRIM65 inhibited LATS1 degradation in TNBC cells over time, thus increasing LATS1 protein expression, indicating that TRIM65 may be involved in the ubiquitination degradation of LATS1. In addition, endogenous LATS1 ubiquitination was reduced in MDA-MB-231 and MDA-MB-453 cells in the sh-TRIM65 group compared with the NC group, and LAST1 protein expression was increased. Furthermore, the results showed that LATS1 protein was degraded by TRIM65 through ubiquitination, thereby reducing LATS1 expression. The above results demonstrate that TRIM65 is upregulated in TNBC, and TRIM65 degrades LATS1 protein expression through ubiquitination.

Several previous studies have found that LATS1 is expressed in various tumors [28–30], and LATS1 has a binding site with E3 ubiquitinating ligase and is targeted by E3 ubiquitin ligase. Ultimately, downregulated expression of LATS1 can alleviate the proliferation, invasion, and migration ability induced by sh-TRIM65 in TNBC. Our results showed that TRIM65 knockdown inhibited the proliferation, invasion, and migration of TNBC cells, and partial proliferation, invasion, and migration of TNBC cells were recovered after further LATS1 knockdown. Taken together, our results indicate that TRIM65 elevated the invasion and migration ability by targeting LATS1 degradation in TNBC.

In conclusion, our results showed that TRIM65 is significantly upregulated in TNBC. TRIM65 holds the capacity for cell proliferation, invasion, and migration of TNBC cells by targeting the ubiquitination and degradation of LATS1. In summary, we have conducted research using clinical specimens, molecules, cells, and animal models to clarify the molecular mechanism of the interaction between TRIM65 and LATS1 to promote TNBC cell proliferation, invasion, and migration. Our findings provide a theoretical and experimental basis for defining a treatment strategy based on TRIM65 gene therapy for TNBC.

The present study has several limitations. First, the binding site of TRIM65 and LATS1 remains unknown, and further ubiquitination degrades LATS1 expression, which needs to be further studied in truncation and mutation experiments. Second, our study focused on the ubiquitin degradation of LATS1 and did not involve the downstream pathway.

## 5. Conclusion

Our results verified that TRIM65 expression is upregulated *in vivo* and *in vitro* and promotes the occurrence and development of TNBC by promoting the invasion and metastasis of TNBC cells. Mechanically, TRIM65 degrades LATS1 expression through ubiquitination, thereby promoting the invasion and metastasis of TNBC cells. These findings suggest that TRIM65 is a potential therapeutic target for TNBC and may play an important role as a new oncogene in TNBC.

## Figures and Tables

**Figure 1:** TRIM65 is upregulated and is an independent risk factor for the prognosis of TNBC. (a) The expression of TRIM65 mRNA. (b) The overall survival of TRIM65 expression in TNBC patients. (c, d) Univariate and multivariate Cox regression analyses of TNBC patient's prognosis. *p* < 0.05, *p* < 0.01, and *p* < 0.001 were considered statistically significant.

**Figure 2:** TRIM65 is upregulated in TNBC. (a, b) Analysis of IHC and representative images showing for TRIM65 expression. (c) Expression of TRIM65 by WB in TNBC patients. (d) Expression of TRIM65 by WB in TNBC from whole lysates of MCF-10A, BT-549, MDA-MB-231, and MDA-MB-453 cell lines. *p* < 0.05, *p* < 0.01, and *p* < 0.001 were considered statistically significant.

**Figure 3:** TRIM65 promotes the malignant biological behavior in vitro. (a, b) The efficiency of lentiviral constructs was measured by RT-qPCR and WB. (c, d) Cell proliferation transfected with sh-TRIM65 or control was assessed by the CCK-8 assay and colony-forming assay in MDA-MB-231 and MDA-MB-453 cells. (e) Representative images and analysis of cell migration and invasion assays in MDA-MB-231 and MDA-MB-453 cells. *p* < 0.05, *p* < 0.01, and *p* < 0.001 were considered statistically significant.

**Figure 4:** TRIM65 promotes cell proliferation *in vivo*. (a) Subcutaneous xenograft tumor model to study the effect of TRIM65 on TNBC. (b–d) Knockdown of TRIM65 reduces tumor weight and volume in mice. (e) H&E staining. (f) Ki67 staining of subcutaneous xenograft tumors. *p* < 0.05, *p* < 0.01, and *p* < 0.001 were considered statistically significant.

**Figure 5:** Expression of TRIM65 is negatively correlated with LATS1. (a) Other proteins were differentially expressed after sh-TRIM65 expression by LC-MS. (b) Correlation expression of TRIM65 with LATS1 and LATS2 based on StarBase database. (c) Knockdown of TRIM65 increased expression of LATS1 but not LATS2 in MDA-MB-231 and MDA-MB-453 cell lines. *p* < 0.05, *p* < 0.01, and *p* < 0.001 were considered statistically significant.

**Figure 6:** TRIM65 accelerates ubiquitin-mediated LATS1 protein degradation. (a) qRT-PCR results of LATS1 mRNA expression in MDA-MB-231 and MDA-MB-453 cells. (b) Co-IP demonstrated the binding of TRIM65 and LATS1 in MDA-MB-231 and MDA-MB-453 cells. (c) WB analysis and CHX release profiles of LATS1 proteins in cells treated with CHX (20 *μ*g/mL) for 0, 2, 4, or 6 hours. (d) WB analysis of ubiquitination assays. *p* < 0.05, *p* < 0.01, and *p* < 0.001 were considered statistically significant. *p* > 0.05 was expressed by n.s.

**Figure 7:** TRIM65 promotes the malignant biological behavior by degrading the expression of LATS1 in TNBC cells. (a, b) Cell proliferation was assessed by the CCK-8 assay and colony-forming assay in MDA-MB-231 and MDA-MB-453 cells. (c) Representative images and analysis of cell invasion and migration assays in MDA-MB-231 and MDA-MB-453 cells. (d) Scientific hypothesis diagram. *p* < 0.05, *p* < 0.01, and *p* < 0.001 were considered statistically significant. ^∗^*p* < 0.05, ^∗∗^*p* < 0.01, and ^∗∗∗^*p* < 0.001.

## Data Availability

All data used to support the findings in the article are available from the corresponding author.

## Abbreviations

TRIM65: Tripartite motif containing 65
TNBC: Triple-negative breast cancer
LATS1: Large tumor suppressor kinase 1
ER: Estrogen receptor
PR: Progesterone receptor
HER2: Human epidermal growth factor receptor 2
Co-IP: Coimmunoprecipitation
CHX: Cycloheximide
shRNA: Short hairpin RNA
sh-TRIM65: Against TRIM65
LC-MS/MS: Liquid chromatography with tandem mass spectrometry
IHC: Immunohistochemical
H&E: Stained with hematoxylin and eosin
RT-qPCR: Quantitative real-time PCR
WB: Western blot
IHC: Immunohistochemical
CCK-8: Cell Counting Kit-8
NC: Negative control
SDS-PAGE: Sulfate polyacrylamide gel electrophoresis
TCGA: The Cancer Genome Atlas
LATS2: Large tumor suppressor kinase 2.

## References

[1] Sung H., Ferlay J., Siegel R. L. (2021). Global cancer statistics 2020: GLOBOCAN estimates of incidence and mortality worldwide for 36 cancers in 185 countries. *CA: a Cancer Journal for Clinicians*.

[2] Li Y., Zhan Z., Yin X., Fu S., Deng X. (2021). Targeted therapeutic strategies for triple-negative breast cancer. *Frontiers in Oncology*.

[3] Boyle P. (2012). Triple-negative breast cancer: epidemiological considerations and recommendations. *Annals of Oncology*.

[4] Cheng M., Liu P., Xu L. X. (2020). Iron promotes breast cancer cell migration via IL-6/JAK2/STAT3 signaling pathways in a paracrine or autocrine IL-6-rich inflammatory environment. *Journal of Inorganic Biochemistry*.

[5] Fang W., Liao C., Shi R. (2021). ZHX2 promotes HIF1*α* oncogenic signaling in triple-negative breast cancer. *eLife*.

[6] Korde L. A., Somerfield M. R., Carey L. A. (2021). Neoadjuvant chemotherapy, endocrine therapy, and targeted therapy for breast cancer: ASCO guideline. *Journal of Clinical Oncology*.

[7] Xin Y., Shen G., Zheng Y. (2021). Immune checkpoint inhibitors plus neoadjuvant chemotherapy in early triple-negative breast cancer: a systematic review and meta-analysis. *BMC Cancer*.

[8] Morreale F. E., Walden H. (2016). Types of ubiquitin ligases. *Cell*.

[9] Tang T., Li P., Zhou X. (2021). The E3 ubiquitin ligase TRIM65 negatively regulates inflammasome activation through promoting ubiquitination of NLRP3. *Frontiers in Immunology*.

[10] Fornage M., Debette S., Bis J. C. (2011). Genome-wide association studies of cerebral white matter lesion burden: the CHARGE consortium. *Annals of Neurology*.

[11] Wang X.-L., Shi W.-P., Shi H.-C. (2016). Knockdown of TRIM65 inhibits lung cancer cell proliferation, migration and invasion: a therapeutic target in human lung cancer. *Oncotarget*.

[12] Yang Y.-F., Zhang M.-F., Tian Q.-H., Zhang C. Z. (2017). TRIM65 triggers *β*-catenin signaling via ubiquitylation of Axin1 to promote hepatocellular carcinoma. *Journal of Cell Science*.

[13] Wei W.-S., Chen X., Guo L.-Y. (2018). TRIM65 supports bladder urothelial carcinoma cell aggressiveness by promoting ANXA2 ubiquitination and degradation. *Cancer Letters*.

[14] Hu G., Liu N., Wang H., Wang Y., Guo Z. (2019). LncRNA LINC01857 promotes growth, migration, and invasion of glioma by modulating miR-1281/TRIM65 axis. *Journal of Cellular Physiology*.

[15] Chen D., Li Y., Zhang X. (2019). Ubiquitin ligase TRIM65 promotes colorectal cancer metastasis by targeting ARHGAP35 for protein degradation. *Oncogene*.

[16] Wu Y.-T., Ma S.-Y., Sun W.-Q. (2021). TRIM65 promotes invasion of endometrial stromal cells by activating ERK1/2/C-myc signaling via ubiquitination of DUSP6. *The Journal of Clinical Endocrinology and Metabolism*.

[17] Ding Y., Chen X., Liu C. (2021). Identification of a small molecule as inducer of ferroptosis and apoptosis through ubiquitination of GPX4 in triple negative breast cancer cells. *Journal of Hematology & Oncology*.

[18] Kim Y.-J., Zhao Y., Myung J. K., Yi J. M., Kim M.-J., Lee S.-J. (2021). Suppression of breast cancer progression by FBXL16 via oxygen-independent regulation of HIF1*α* stability. *Cell Reports*.

[19] Guo Y., Li Q., Zhao G. (2021). Loss of TRIM31 promotes breast cancer progression through regulating K48- and K63-linked ubiquitination of p53. *Cell Death & Disease*.

[20] Zhou C., Zhang Z., Zhu X. (2020). N6-Methyladenosine modification of the TRIM7 positively regulates tumorigenesis and chemoresistance in osteosarcoma through ubiquitination of BRMS1. *eBioMedicine*.

[21] Lim J.-E., Choi B., Jee S. H. (2020). Urinary bisphenol A, phthalate metabolites, and obesity: do gender and menopausal status matter?. *Environmental Science and Pollution Research International*.

[22] Jia J., Jin J., Chen Q. (2020). Eukaryotic expression, Co-IP and MS identify BMPR-1B protein-protein interaction network. *Biological Research*.

[23] Meroni G., Desagher S. (2022). Cellular function of TRIM E3 ubiquitin ligases in health and disease. *Cell*.

[24] Haque S., Cook K., Sahay G., Sun C. (2021). RNA-based therapeutics: current developments in targeted molecular therapy of triple-negative breast cancer. *Pharmaceutics*.

[25] Lang X., Tang T., Jin T., Ding C., Zhou R., Jiang W. (2017). TRIM65-catalized ubiquitination is essential for MDA5-mediated antiviral innate immunity. *The Journal of Experimental Medicine*.

[26] Wu S.-Y., Xiao Y., Wei J.-L. (2021). MYC suppresses STING-dependent innate immunity by transcriptionally upregulating DNMT1 in triple-negative breast cancer. *Journal for Immunotherapy of Cancer*.

[27] Li T., Tao Z., Zhu Y. (2021). Exosomal annexin A6 induces gemcitabine resistance by inhibiting ubiquitination and degradation of EGFR in triple-negative breast cancer. *Cell Death & Disease*.

[28] Tang F., Gao R., Jeevan-Raj B. (2019). LATS1 but not LATS2 represses autophagy by a kinase-independent scaffold function. *Nature Communications*.

[29] Pan W.-W., Moroishi T., Koo J. H., Guan K.-L. (2019). Cell type-dependent function of LATS1/2 in cancer cell growth. *Oncogene*.

[30] Kazimierczak U., Dondajewska E., Zajaczkowska M., Karwacka M., Kolenda T., Mackiewicz A. (2021). LATS1 is a mediator of melanogenesis in response to oxidative stress and regulator of melanoma growth. *International Journal of Molecular Sciences*.

